The article "IoT Based System for Heart Monitoring and Arrhythmia Detection Using Machine Learning" was published in 2023. Journal: J Healthc Eng.

# IoT Based System for Heart Monitoring and Arrhythmia Detection Using Machine Learning

**DOI:** 10.1155/2023/6401673

**Published:** 2023-02-08

**Authors:** Ruben Enrique Cañón-Clavijo, Carlos Enrique Montenegro-Marin, Paulo Alonso Gaona-Garcia, Johan Ortiz-Guzmán

**Affiliations:** ^1^Faculty of Engineering, Universidad Distrital Francisco José de Caldas, Bogotá, Colombia; ^2^Fundación Universitaria Internacional el Rioja, Bogotá, Colombia

## Abstract

Internet of Things (IoT) technologies allow building a digital representation of people, objects, or physical phenomena to be available on the Internet. Thus, stakeholders can access this information from remote places or computational systems could analyze this data to find patterns, make decisions, or execute actions. For instance, a doctor could diagnose patients by analyzing the received data from an IoT system even when patients are located in a remote place. This article proposes an IoT system for monitoring electrocardiogram (ECG) signal and processing heart data in order to generate an alert when an arrhythmia is present. This system involves a Polar H10 heart sensor, machine-learning models to classify heart events, and communication technology to share and store patient's information. In the first place, the architecture of the IoT monitoring system and the communication between the components are described by discussing the designing criteria. Second, the experimentation process performs the training and the assessment of three classification algorithms, random forest, convolutional neural network, and k-nearest neighbors. The results show that k-nearest neighbor has the best accuracy percentage classifying the arrhythmias under study (premature ventricular contraction 94%, fusion of ventricular beat 81%, and supraventricular premature beat 82%); also, it is able to discern normal and unclassifiable beats with 93% and 97%, respectively.

## 1. Introduction

The Internet of Things and artificial intelligence are emergent fields where researchers are developing methods and techniques to reduce human effort [1, 2]. While IoT is relying on communication technology, sensors, and data processing technics [3]; classification algorithms are used to recognize a hidden pattern in the input data and identify the class where it belongs [4].

It is possible to apply this technology in fields such as industry, farming, meteorology, or medicine. For instance, a medical cyber-physical system (MCPS) is a concept where software, sensors, and networks interacting with physical human signals in order to improve the effectiveness of the patient's medical care. In this way, sensors capture biological signals and send them through a network to be processed by software algorithms that extract useful information and take actions, such as emitting an alert, diagnosis, or even providing treatment in order to easily improve the patient's health care [5]. Due to the high costs associated with in-hospital care, alternatives including home care, assisted living, telemedicine, and sport-activity monitoring, have drawn more interest. Likewise, mobile monitoring and home monitoring of vital signs and physical activities allow health to be assessed remotely at all times [5].

The article "IoT Based System for Heart Monitoring and Arrhythmia Detection Using Machine Learning" was published in 2023. Journal: J Healthc Eng.

On the other hand, according to the World Health Organization, cardiovascular disease is the leading cause of death with an estimated 32% of all deaths worldwide [6]. Similarly, sudden cardiac death (SCD) and arrhythmia represent between 15% and 20% of all deaths in the world.

Sometimes arrhythmias are detected when complications appear; knowledge of the characteristic ECG changes may provide early clues to the presence of these disorders, the prompt recognition of which can be lifesaving [7]. Therefore, continuous heart monitoring is required for early detection in order to give a suitable treatment for patients with cardiac arrhythmias [8].

In order to detect and diagnose heart diseases, the electrocardiogram (ECG) is an indispensable tool for monitoring the electrical activity of the heart [9]. The ECG has allowed for studying and classifying different arrhythmias types according to their particular characteristics. Based on this typology, different studies have proposed using machine learning in order to extract ECG data patterns for the early identification of arrhythmias. In this way, machine learning algorithms such as k-nearest neighbors (KNN), convolutional neural networks (CNNs), and random forest has shown interesting result in arrhythmia classification [10–12].

In this work, we propose a system for monitoring the patient's heart signal and analyzing the heart data by using machine learning for detecting arrhythmias. Thus, when the machine-learning algorithm detects an arrhythmia, it generates an alert. In order to allow caretakers to see the patient's heart activity, the system provides a web application that displays the ECG chart and the generated alerts.

For capturing the heart signal, the Polar H10 heart monitor is selected because of its good performance [13]. In addition, it provides an ECG sensor and software necessary for accessing the captured data and sending it to the mobile terminal (via Bluetooth). This last, send the heart data through the message broker, which delivers the published data to the classification component.

The classification component includes a classification algorithm selected by testing three classification algorithms (CNN, KNN, and random forest) and assessing their performance. It is in charge of receiving the heart data and recognizing patterns in order to classify the input data as arrhythmia (premature ventricular contraction, fusion of ventricular beats, or supraventricular premature beats) or normal beats. If the input data are an arrhythmia, the system generates an alert to avoid complications in the patient's health.

The article "IoT Based System for Heart Monitoring and Arrhythmia Detection Using Machine Learning" was published in 2023. Journal: J Healthc Eng.

The goal of this IoT system is to improve the medical care service to people at potential risk for heart incidents located at remote places by providing a monitoring system that helps doctors in the patient's heart signal supervision. Besides, authorized people can supervise patients accessing their ECG via the web.

The remainder of the article is organized as follows: Section 2 introduces previous works in reference to cardiovascular disease prediction and supervision systems based on IoT.  Section 3 describes the MIT-Arrhythmia database used for training the classifier models.  Section 4 shows the system's architecture describing each component proposed.  Section 5 presents the experimentation for building the classification model.  Section 6 presents the results and discussion. Finally, Section 7 resumes the considerations and conclusions of the work.

## 2. Related Work

Interest in machine learning applications such as health care and medical science is growing considerably [14]. For instance, Ellaji et al. design an architecture of a narrowband IoT system to integrate wearable devices to improve medical health care. The main benefits of using narrowband IOT are its low and low power consumption. Therefore, it provides a novel mechanism for linking all the smart devices, which requires a very less amount of data and long-range intervals. This improves hospital data transmission and accomplishes data processing in real time. The narrowband IoT system includes an application server, NB-IoT devices, cloud stage, and customer applications. First, NB-IoT devices send sensing data to the cloud platform and it stores the data. Different applications process data subsequently clients can access this information through a user interface [15].

Ahamed et al. [16] propose a cardiovascular disease prediction system applying five machine-learning algorithms (random forest, decision tree, Naive based, k-nearest neighbors, and support vector machine). Their methodology includes four tiers as follows:

1. Data collection: tier 1 collects data from IoT sensors or wearables devices using ThingSpeak Cloud, which is an Internet of things analytics service that allows aggregating, visualizing, and analyzing live data streams in the cloud [17].
2. Data storage: tier 2, preprocesses and stores data using Heroku's PostgreSQL cloud, an open-source database as a service that provides a trusted, secured, and scalable storage platform [18].
3. Data Analysis on a cloud: this tier uses different machine learning models to predict the output class for heart input data. They choose the model based on the best performance.
4. User interface: this tier provides a graphical user interface to allow doctors and patients to access clinical results.

The article "IoT Based System for Heart Monitoring and Arrhythmia Detection Using Machine Learning" was published in 2023. Journal: J Healthc Eng.

The work [19] presents an architecture of an embedded platform for web-based monitoring and medicine schedule reminder. This platform allows patients and health professionals to access the data captured by the sensor through a web monitoring system and it generates an alert according to the medicine schedule. Sensors transmit data through ZigBee or Bluetooth to manage units and RFID allows linking patient records with unique identification numbers. Additionally, they use the MQTT protocol to share data between components.

Barbosa et al. designed a telemonitoring system for patients with cardiovascular disease [20]. This system allows caretakers to monitor the signals and symptoms of patients with heart disease while patients reside at home, in this sense, telemonitoring means monitoring from a remote place. On the other hand, this system follows the continua design guidelines (CDG) in order to provide security to medical data flow among sensors, gateways, and health information services. The CDG is an open framework for secure and interoperable health data exchange in personal connected health. The CDG provides a set of clearly defined interfaces that enable the secure flow of medical data among sensors, gateways, and end services, removing ambiguity in underlying standards to ensure a consistent and interoperable ecosystem of personal connected health devices [21].

Heart and breath data are telemonitoring in the system presented in [22]. A DatascopeTrio acquires heartbeat and breathing frequency then this data are stored in a database and a JSP-based web allows clients to monitor patient's data.

Works as [23] present a self-diagnosis system of cardiovascular disease based on IoT. Sensors transmit the data to an Android application via Bluetooth then, the application stores this data using a CRUD REST API. Finally, the heart rate data are analyzed using the theory of probability. The previous system is used for studying stress' effects on cardiac dynamics [24].

## 3. Background

As follows, some necessary concepts and backgrounds related to ECG, arrhythmias, IoT, and machine learning are presented.

### 3.1. Electrocardiogram

Electrocardiogram (ECG) lead is a recording of the heart's electrical activity. Therefore, a 12-lead ECG is a recording of cardiac electrical activity from 12 different perspectives [25]. This ECG configuration builds up a three-dimensional characterization of the heart's electrical activity.

The article "IoT Based System for Heart Monitoring and Arrhythmia Detection Using Machine Learning" was published in 2023. Journal: J Healthc Eng.

Figure 1. Shows the twelve lead groups, on the right the frontal leads, and the transverse leads on the right.

Vertical plane (frontal leads): six frontal leads provide information about the heart's vertical plane: lead I, lead II, lead III, augmented vector right (aVR), augmented vector left (aVL), and augmented vector foot (aVF). In this configuration, three electrodes are placed on the right arm, the left arm, and the left leg. Given the electrode placements, these leads detect electrical activity in the frontal plane.

Horizontal plane (transverse leads): this configuration provides information about the heart's horizontal plane: V1, V2, V3, V4, V5, and V6. On the right side of Figure 1, is the localization of the electrodes of transverse leads. The transverse leads are unipolar and require only a positive electrode, the negative pole of all 6 leads is found at the center of the heart [27].

#### 3.1.1. Modified Limb Lead

During exercise stress testing, the motion of the limbs can disrupt the ECG recordings and in conditions where limbs become clinically inaccessible, the modified limb electrode position on the torso addresses the above problem [28]. In the modified limb lead (MLL) configuration, the right arm electrode is placed on the subject's third right intercostal space, slightly to the left of the midclavicular line. The left arm electrode is placed in the fifth right intercostal space, slightly to the right of the midclavicular line, and the left leg electrode is placed in the fifth right intercostal space, on the midclavicular line [29].

#### 3.1.2. Ambulatory ECG

Ambulatory ECG (AECG) devices allow the cardiac rhythm to be monitored and recorded over days, weeks, or years and are used primarily in the outpatient setting [30]. Recording may take place continuously or occur intermittently in response to patient activation or auto-sensing of rhythm disturbances. Multiple devices are available, being the Holter monitors, ambulatory telemetry monitors (ATMs), and patch electrode monitors (PEMs) are the most common [31]. Other ambulatory ECGs include an event monitor, external loop monitor, implantable loop monitor, and pacemaker [32].

### 3.2. Cardiac Arrhythmia

Cardiac arrhythmias are disturbances in the rhythm of the heart, manifested by abnormally fast or slow rates [33]. Sinus rhythm represents the heart's normal rhythm and its rate is between 60 and 100 beats per minute (bpm) while you are resting. Sinus bradycardia occurs when the sinus rhythm is slower than 60 bpm, and if the sinus rhythm is faster than 100 bpm, it is called sinus tachycardia [34].

The article "IoT Based System for Heart Monitoring and Arrhythmia Detection Using Machine Learning" was published in 2023. Journal: J Healthc Eng.

The typical arrhythmia symptoms include palpitations (being aware of your heartbeat), weakness, shortness of breath, lightheadedness, dizziness, fainting (syncope), and, occasionally, chest pain. The symptoms tend to be more severe when the rate is faster. However, sometimes there are no symptoms, and the condition is evident during a routine examination. A tachyarrhythmia that is rapid enough and lasts long enough can produce cardiomyopathy and congestive heart failure. In these cases, treatment of the arrhythmia can often return normal function to the ventricles. Although certain physical signs present during arrhythmias can help the physician make a correct diagnosis, electrocardiography is the standard method used for recognizing cardiac arrhythmias [33].

Typical sinus bradycardia causes are as follows:

- Medicines such as beta-blockers, including eye drops, which contain beta-blockers
- An underactive thyroid gland
- Hypothermia
- Tachy-brady syndrome

Typical sinus tachycardia causes are as follows:

- Underlying health conditions such as an overactive thyroid gland
- Severe anemia
- Infections
- Severe blood loss
- Stimulants such as caffeine, nicotine, and alcohol
- Prescribed medicines such as salbutamol
- Illegal drugs such as amphetamines, cocaine, ecstasy, and cannabis

#### 3.2.1. Arrhythmia Types

There are many different types of arrhythmia; the type depends on where the rhythm starts in the heart, and whether the heartbeat is too fast, or too slow.

Premature heartbeat: A premature, or extra, beat is a common, usually harmless type of arrhythmia that typically does not cause symptoms. Most healthy people who experience an occasional extra beat do not need treatment. However, a premature heartbeat can lead to a longer-lasting arrhythmia in persons with previous heart disease.

Supraventricular arrhythmias (SVT): these arrhythmias are tachycardias that start from above the ventricles. SVTs are quite common and rarely life-threatening.

The principal types of supraventricular arrhythmias include [35]the following:

Inappropriate sinus tachycardia: this is a fast heart rhythm, which can happen suddenly, with no obvious cause. While resting, the heart rate can quickly rise to over 100 bpm and with a very small amount of activity; it can quickly rise to 150 bpm. It is more common in young women [34].

Atrial fibrillation (AF): this happens when many impulses begin and spread through the atria. This results in a disorganized rapid and irregular rhythm. Because the impulses are traveling through the atria in a disorderly fashion, there is a loss of coordinated atrial contraction.

The article "IoT Based System for Heart Monitoring and Arrhythmia Detection Using Machine Learning" was published in 2023. Journal: J Healthc Eng.

Atrial flutter: an atrial arrhythmia caused by one or more rapid circuits in the atrium. Atrial flutter is usually more organized and regular than atrial fibrillation.

Supraventricular premature beats (SPB): these represent premature activation of the atria from a site other than the sinus node and can originate from the atria or the atrioventricular node, though the vast majority are atrial in origin. Atrial premature beats (APBs) are also referred to as atrial premature complexes, premature atrial beats, and premature atrial complexes. This includes patients without structural heart disease and those with any form of cardiac disease, independent of severity [36].

Ventricular Arrhythmias: ventricular arrhythmias are fast, abnormal heart rhythms that start from the ventricles. Most ventricular arrhythmias are caused by underlying heart disease, and can often be life-threatening [35]. Types of ventricular arrhythmias include.

Fusion beats: it is the presence of fusion beats, which identify simultaneous depolarization of the ventricle by both the normal conduction system and an ectopic impulse originating in the ventricle.

A fusion beat occurs when electrical impulses from different sources act upon the same region of the ventricular chambers at the same time.

Premature ventricular contractions (PVCs): they are early, extra heartbeats that start out in the ventricles. Most of the time, PVCs do not cause any symptoms or require treatment [35].

Ventricular tachycardia (VT): it is a rapid heartbeat that begins in the ventricles. The rapid rhythm keeps the heart from adequately filling with blood, and less blood is able to pump through the body. VT can be serious, especially in people with heart disease, and may be associated with more symptoms than other types of arrhythmia.

Ventricular fibrillation (VF): it is an erratic, disorganized firing of impulses from the ventricles. The ventricles quiver and cannot generate an effective contraction, which results in a lack of blood being delivered to your body.

### 3.3. Medical Cyber-Physical System

Medical cyber-physical systems (MCPS) are the combination of embedded software controlling devices, networking capabilities, and the complicated physical dynamics of the human body in order to improve the effectiveness of medical care by monitoring patients' physical signals and providing proper treatment while ensuring safety [5]. Depending on their main functionality, it is possible to categorize the MCPS devices into two large groups as follows:

- Monitoring devices: they provide different kinds of clinic-relevant information about patients such as heart rate, oxygen level, blood pressure, and temperature
- Delivery devices: they provide an actuate therapy in order to change the patient's physiological state

In MCPS, interconnected monitoring devices can feed collected for decision support. For example, caregivers can analyze the information provided by monitoring devices and then use delivery devices to initiate treatment. In order to illustrate applications of MPCS examples are presented as follows:

Pumps are commonly used to deliver opioids for pain management but patients have different reactions to the medications and require distinct dosages and delivery schedules. A major problem with opioid medications in general is that an excessive dose can cause respiratory failure. An MCPS can be designed to deliver the doses according to the patient's profile in order to prevent an overdose. Additionally, it can monitor the oxygen level, if some complication appears it can emit an alert.

The article "IoT Based System for Heart Monitoring and Arrhythmia Detection Using Machine Learning" was published in 2023. Journal: J Healthc Eng.

Sometimes is necessary to take X-ray images during surgical procedures under general anesthesia. During the procedure, the patient breathes with the help of a ventilator. Because patients on ventilators cannot hold their breath to avoid blur in the X-ray image caused by moving lungs, the ventilator has to be paused and later restarted. In some unfortunate cases, the ventilator is not restarted, leading to the death of the patient. A safer alternative is to let the ventilator transmit its internal state to the X-ray machine. In this approach, the X-ray machine receives the state of the breathing cycle in order to decide the convenient instance when it can take an X-ray image [5].

### 3.4. MQTT Protocol

MQTT is a client-server publish/subscribe messaging transport protocol. It is lightweight, open, simple, and designed to be easy to implement. These characteristics make it ideal for use in many situations, including constrained environments such as for communication in machine-to-machine and Internet of Things (IoT) contexts.

The protocol runs over TCP/IP, or over other network protocols that provide ordered, lossless, bi-directional connections. Its features include; the use of the publish/subscribe message pattern providing one-to-many message distribution and decoupling of applications [37].

Client: a program or device that uses MQTT and always establishes the network connection to the server.

Server: a program or device that acts as an intermediary between clients, which publish application messages, and clients, which have made subscriptions.

Topic Name: it is the label attached to an application message, which matches the subscriptions known to the server. The server sends a copy of the application message to each client that has a matching subscription [37].

The article "IoT Based System for Heart Monitoring and Arrhythmia Detection Using Machine Learning" was published in 2023. Journal: J Healthc Eng.

**EMQX** is an open-source MQTT broker with a high-performance real-timemessage-processing engine, powering event streaming for IoT devices at a massive scale [38].

The benefits of EMQX broker are as follows:

- Massive Scale: scale to 100 million concurrent MQTT connections with a single cluster
- High performance: move and process millions of MQTT messages per second in a single broker
- Low latency: guarantee submillisecond latency in message delivery with the soft real-time runtime
- High scalability, security, and reliability

### 3.5. JavaScript Object Notation

**JavaScript Object Notation (JSON):** is a lightweight data-interchange format. It is written as such a property list enclosed in braces ({}), with name-value pairs separated by commas (), and with the name and value of each pair separated by a colon (). In JSON each property name and each string value must be enclosed in double quotation marks (“) [39].

The benefits of JSON are as follows:

- JSON is a text format completely language independent
- It is easy for humans to read and write
- It is easy for machines to parse and generate

### 3.6. Machine Learning

Machine learning has three main learning approaches, supervised learning, unsupervised learning, and reinforcement learning [40]. The most general problem approachable by a supervised method is predicting a variable (answer or label) when some others (predictors) are known. As an example, in medical diagnosis, the predictors could be clinical parameters such as temperature, blood pressure, and cholesterol, and the answer could be the knowledge if the patient is sick or not.

Supervised learning includes a first stage called training, where the predictors and the answer (labeled data) are provided letting the system learn how to find an answer based on the predictors. If the training is successful, the algorithm is able to automatically predict the answer for any other datasets including the same predictors [41].

Some remarkable supervised learning algorithms are the decision tree, random forest, logistic regression, and KNN [42]. Regarding this project, the following algorithms are used:

#### 3.6.1. Convolutional Neural Network

Convolutional neural network (CNN) is a deep learning model for handling information that has a grid pattern, such as images; however, they are also efficient with audio data, temporal series, and signals. This algorithm learns spatial hierarchies of features, from low-to-high-level patterns. CNN has typically three types of layers, convolution, pooling, and fully connected. The convolutional layer is responsible for extracting features from the data, while the polling layer is in charge of reducing the dimensionality of the feature map keeping the essential elements. Once the features extracted by the convolution layers and downsampled by the pooling layers are created, they are mapped by a subset of fully connected layers to the final outputs of the network (classes) [43].

The article "IoT Based System for Heart Monitoring and Arrhythmia Detection Using Machine Learning" was published in 2023. Journal: J Healthc Eng.

The advantages of CNN are as follows:

- It automatically detects important features without any human supervision
- High accuracy in image recognition and classification
- CNN is computationally efficient by minimizing computation operations

#### 3.6.2. K-Nearest Neighbors

The classification approach of K-nearest neighbors [44] is an instance learning where the algorithm classifies new observations based on the similarity to the rest of the data points stored in the model. The process takes a new observation and selects the K closest points to the new example then selects the most common class between them by the majority vote [45].

The classification has two stages, first determining the nearest neighbors and second, deciding the class based on these neighbors.  Figure 2 illustrates the KNN process: in this case, the algorithm finds the nearest neighbors, three triangles, one circle, and one plus. The majority is for the triangle class with three votes; therefore, the algorithm classifies the element (?) as a triangle class.

The advantages of KNN are as follows:

- It has no training period, it just stores the dataset during the training period and learns from it when performs real-time predictions
- Since the KNN algorithm requires no training before making predictions, new data can be added and this will not affect the accuracy of the algorithm
- Low-complex implementation

#### 3.6.3. Random Forest

The random forests algorithm is a combination of multiple tree predictors where each tree depends on a random vector. This algorithm generates a large number of trees using the training dataset, then they vote for the most popular class [46].

Figure 3 represents a general schema of the random forest process as follows:

Random forest procedure as follows:

- Step 1: select random samples from the training dataset.
- Step 2: build a decision tree for the K data point.
- Step 3: chose the n-tree subset from the generated trees and execute step 1 and step 2.
- Step 4: the final class is the most voted one.
- They also offer a superior method for working with missing data. Missing values are substituted by the variable appearing the most in a particular node. Among all the available classification methods, random forests provide the highest accuracy.

The article "IoT Based System for Heart Monitoring and Arrhythmia Detection Using Machine Learning" was published in 2023. Journal: J Healthc Eng.

The advantages of the random forest are as follows:

- It can handle big data with numerous variables running into thousands
- It can automatically balance data sets when a class is more infrequent than other classes in the data

The method also handles variables fast, making it suitable for complicated tasks.

#### 3.6.4. Confusion Matrix

The confusion matrix is a tool for measuring the performance classification of machine learning models. In addition, we can say confusion matrix is a summarized table of the number of correct and incorrect predictions generated by a classifier.

Table 1 represents an example of a confusion matrix as follows:

- True Positive (TP): the actual value was positive and the model predicted a positive value
- False Positive (FP): the prediction is positive, and it is false
- False Negative (FN): the prediction is negative, and the result is also false
- TN: True Negative: the actual value was negative and the model predicted a negative value

Accuracy is a measure of how many correct predictions the model made for the complete test dataset. This is a convenient metric to evaluate the performance of classification models [47].

## 4. MIT-BIH-Arrhythmia Database

The MIT-BIH-Arrhythmia database is a set of standard test materials for the evaluation of arrhythmia detectors. These detectors are algorithms that identify normal or abnormal signals by using detection or classification techniques [48]. The MIT-BIH-Arrhythmia is a convenient testing dataset since it provides a variety of and well-characterized arrhythmia data [49].

This database contains samples of two-channel ambulatory ECG recordings, obtained from 47 subjects studied by Boston's Beth Israel Hospital Laboratory. In most records, one channel is a modified limb lead II (MLII), obtained by placing the electrodes on the chest. and the other channel is usually V1 and, to a lesser extent, V2, V4, or V5 [50]. This work takes samples of five classes from the MIT-BIH-Arrhythmia database as follows:

- *N*: normal beat
- *S*: supraventricular premature beat
- *V*: premature ventricular contraction
- *F*: fusion of ventricular and normal beat
- *Q*: unclassifiable beat

## 5. System Architecture

This section presents the architectural design decisions to accomplish the requirements of the system. In this sense, four components interoperate to capture and process data to present useful information to the user, as shown in Figure 4.

**Sensing manager:** it is a mobile application that manages the sensing data that the ECG sensor sends via Bluetooth.

**CRUD REST API:** it provides create, read, update, and delete operations to other components in order to exchange information with the database.

The article "IoT Based System for Heart Monitoring and Arrhythmia Detection Using Machine Learning" was published in 2023. Journal: J Healthc Eng.

**Monitoring GUI:** it is a web application where users can access for monitoring patients through a graphic user interface.

**Data structures:** in order to exchange information between components, every data structure is defined in JSON format given the benefits of easy parsing and reading data.

**Data exchange:** a message broker allows sharing between components.

### 5.1. Sensing Component

The Polar H10 ECG sensor captures the heart data and sends it to a mobile application via Bluetooth [13]. The mobile application integrates the Polar SDK [51], which provides libraries to interpret the coming data. Once, the data are available in the mobile application, it is transformed into a JSON message, Table 1, in order to publish in an MQTT topic. The following data are sent to the MQTT server:

- ECG: ECG data array
- Date: current timestamp
- PatientId: patient identifier

### 5.2. Message Broker

In order to share data between components, the message broker intermediates the data exchange by publishing/subscribing to data on topics. For instance, the monitoring component and detection component subscribe to the heart data topic; when the sensing component publishes data on a given topic the message broker sends it to subscribers. The message broker enables the integration of components without coupling.

Coupling is an undesirable interdependence between components or modules. It is suitable in software design to keep low coupling because it allows making changes in one component without affecting the others.

Given the performance of the EMQX broker for IoT devices, it is selected to manage the message exchange in the system.

### 5.3. Data Storage

All data needed by the system is stored on a document database due to its capability of storing data structures such as JSON directly. This means it is not required to transform the JSON element data because document databases store data as JSON documents, instead of columns as needed by a relational database. This feature eases the data persistence implementation.

Patients' personal data (id and names), heart data events (id, ECG, and timestamps), and medical staff data (id, names, and credentials) are represented in JSON format.

### 5.4. CRUD Component

The purpose of the REST API is to provide the required CRUD operations (create, read, update, and delete) on the database. This implies just API REST has direct communication with the database; therefore, every component that needs to exchange data with the database has to do it by sending HTTP requests to the REST API. In this way, every component has to implement a REST client to use the operation that REST API exposes. The detail of the CRUD operations are as follows:

**Create operation:** the API provides endpoints for saving heart incidents when arrhythmia is detected, for this purpose, the REST client must send this data (patient Id, type of arrhythmia, and timestamp) in the request, and the API saves the register in the database.

The article "IoT Based System for Heart Monitoring and Arrhythmia Detection Using Machine Learning" was published in 2023. Journal: J Healthc Eng.

**Read operation:** the API provides endpoints for reading heart data by sending the patient's Id. In the same way, medical stuff data (name, id, and credentials) are returned when the proper id is sent in the request.

**Update operation:** the API provides endpoints for updating personal data or credentials by sending the proper id and the data to be updated.

**Delete operation:** the API provides endpoints for deleting the register by sending the id. This operation is enabled just to unsubscribe medical stuff.

Although API REST can handle different formats to exchange data, JSON is suitable to meet the need of this system, so all data structures use JSON format.

Given that API REST provides the required operation on the database, all components must implement REST clients to perform these operations instead of implementing database clients it selves. This implies REST API depends on the database implementation but avoids coupling with other components. This means any change in the database implementation affects the API REST but the other components have no impact.

### 5.5. Arrhythmia Detection Component

This component requires a machine learning model to recognize arrhythmia patterns, such as premature ventricular contraction, a fusion of ventricular beat, or supraventricular premature, on the heart data. For this purpose, an experimentation phase is performed in order to evaluate different classification algorithms and select the model with the best performance (see section 7). As a result of this experimentation, the selected model is integrated into the detection component.

The detection component is a subscriber of the heart data published by the sensing component. Therefore, when heart data are published, the MQTT sends it to the arrhythmia detection component. Then, the machine-learning model processes the information and performs the classification. If the algorithm classifies the data as any arrhythmia, the component registers the alert using the proper operation. In this way, API REST creates a new record of heart data incidents in the database.

### 5.6. Monitoring Component

The heart monitor is a web application that provides a graphical user interface where authorized people access patients' data. When a user tries to login into the system by sending his credentials, the web application read the corresponding staff data by using a proper read operation from API REST. If the credentials are correct, the login is valid and the user can access to the system.

The article "IoT Based System for Heart Monitoring and Arrhythmia Detection Using Machine Learning" was published in 2023. Journal: J Healthc Eng.

ECG data are received from the message broker in order to build the ECG chart in real time. Additionally, the alert list is disposed of in the web application; this data are obtained through the proper API REST read operation.

## 6. Experimentation

This section describes the arrhythmia dataset and explains the applied methodology in this work for building and choosing the classification model.

### 6.1. Model Building Process (Offline)

This process split the dataset into two subsets, 70% of the data are for training and 30% for testing; this is a typical proportion used in machine learning [52].

The algorithm learns from the training data where each sample has a feature vector and a known category so the model adjusts its parameters with every sample to improve the classification.

In the next step, the algorithm receives data from the testing group with unknown categories, and the algorithm has to classify each input element in the correct category or class. For measuring the model accuracy, the convolutional matrix is generated. The classification accuracy is represented by the percentage of data labeled in the right category and misclassification take place when samples are classified into categories they do not belong.

Training samples have the same quantity for each class in order to balance the training set as shown in Figure 5.

It is necessary to normalize the sample and take the same number of characteristics in the feature vector. Thereby, 180 features are included and they are normalized between zero and one.

Based on this dataset, three machine-learning algorithms receive this dataset to build the classification models. Then, each model runs tests with the validation data to measure its classification performance. This test gives us the percentage of success and failure in the classification. The model with the best classification performance is selected as a part of the detection component.

### 6.2. Arrhythmia Detection Component

The arrhythmia component integrates the best classification model from the offline process. It receives data from the message broker to process and classify into the five given classes. Each input data corresponds to the output label. When the output label is ventricular, supraventricular, or fusion beat, the component registers an alert in the database using the CRUD component. Unlike the offline building process, the detection process receives incoming data in real time from the MQTT broker.

## 7. Results and Discussion

This section resumes the results and discussion about the main findings for architectural decisions and experimentation.

The article "IoT Based System for Heart Monitoring and Arrhythmia Detection Using Machine Learning" was published in 2023. Journal: J Healthc Eng.

### 7.1. Architectural Decisions

The proposed architecture allows the decoupling of each component of the system keeping the single principle responsibility [53] and they communicate with each other by sharing data in the message broker. This desegregation permits every component to take advantage of different technologies and programming languages, for example, python for data analysis, angular for graphical user interface, and spring boot for the API REST implementation.

By selecting JSON as a format for data exchange allows for simplifying data handling by every component. On the other hand, the document database let the direct storage of data in JSON format and transformation is not necessary.

Finally, instead of connecting directly with the database, every component uses the CRUD operations that API REST provides. This approach simplifies the implementation given every component that needs stored data to have to use the proper API REST operation instead of implementing database connection by itself.

### 7.2. Model Training and Performance Assessment

The classifier model is an essential part of the system because it is in charge of receiving heart data and categorizing in any of the five classes. Thus, errors in classification could lead to a fake alert or hiding real heart incidents so it is necessary to test different classifier models and select the model with the best performance.

The first approach is a convolutional neural network (CNN). The confusion matrix in Figure 6 shows the results of this algorithm. This reveals a high classification accuracy for normal beats, a fusion of ventricular, and unclassifiable beats but low performance for other classes.

CNN classifies 83% of the normal beats correctly but 7% as a fusion of ventricular, 5% as premature ventricular contraction, 3% as unclassified, and 2% as supraventricular. Fusion of ventricular class has 91% of data well classified but 1% are misclassified as ventricular and 9% as normal. Similarly, 89% of unclassified class belongs to the correct category but 9% are labeled as normal and 1% as ventricular.

Instead of previous classes, supraventricular classification has a poor performance, just 48% of data are in the correct category, and almost half of them 47% are misclassified as supraventricular, 2% as ventricular, 3% as fusion beats, and 1% as unclassified. Likewise, Ventricular beats have 61% of accuracy, and 21% are labeled as normal, 2 as supraventricular, 7% as fusion beats, and 9% as unclassified beats.

The most remarkable results are 47% of supraventricular and 21% of ventricular data are classified as normal beats. In practice, the system skips a high number of incidents of these classes so it never registers these events because it considers them as normal beats. For this reason, it is necessary to find a better performance in the classification.

The article "IoT Based System for Heart Monitoring and Arrhythmia Detection Using Machine Learning" was published in 2023. Journal: J Healthc Eng.

The second approach uses a random forest algorithm to perform the classification; Figure 7 shows the confusion matrix. This algorithm improves the classification accuracy for some classes but reduces it for others.

Classification accuracy increases by 9% for normal class and supraventricular. However, accuracy decreases by 8% for fusion beats and 4% for unclassified beats.

Despite a better performance for normal and supraventricular classification, the algorithm reduces accuracy for fusion and unclassified beats.

Focus on the misclassification percentage of supraventricular data, it is remarkable that the reduction of data labeled as normal being supraventricular. It implies this algorithm detects 6% additional incidents of this type but increments by 11% for ventricular, 6% for fusion beats, and 5% for unclassified beats in the percentage of misclassification as normal.

The results show the general performance of the random forest algorithm is worse than the convolutional neural network performance. Therefore, it is not suitable to use this algorithm for this work.

The third approach is a classifier based on k-nearest neighbors, Figure 8. This algorithm achieves a considerable improvement in classification accuracy, especially for normal, supraventricular, and unclassified classes.

It gets 93% of correct classification for normal class reducing the misclassification error as follows: supraventricular 4%, ventricular 2%, fusion beats 1%, and no errors in unclassified.

In regards to supraventricular classification, random forest, and CNN algorithms have problems distinguishing supraventricular samples from normal samples so they reach errors greater than 40%. By contrast, the KNN algorithm gets the best performance in this topic with 82% of accuracy and 13% of data misclassified as normal, 3% as ventricular, 1% as fusion beats, and 0% as unclassified.

KNN has an excellent performance classifying ventricular samples with 94% of accuracy, 33% greater than CNN and random forest results. On the other hand, 2% of ventricular samples are labeled as normal, 1% as supraventricular, 2% as fusion beats, and 1% as unclassified.

The accuracy of KNN classifying fusion beats is worse than CNN and random forest where they have 10% and 2% higher accuracy, respectively, than KNN. This increment of the error is related to 11% of fusion beats samples misclassified in the ventricular class. However, in practice, this behavior is better than having a high percentage in any class of arrhythmia that is considered a normal beat because it implies the system generates no alert.

The article "IoT Based System for Heart Monitoring and Arrhythmia Detection Using Machine Learning" was published in 2023. Journal: J Healthc Eng.

KNN classifies 97% of unclassified samples correctly labeling 2% of them as normal and 1% as fusion beats. This algorithm is able to differentiate perfectly unclassified samples from supraventricular and fusion beats.

Considering all of these, the KNN is the algorithm with the best performance result for this system; it improves the lowest scores obtained by CNN and random forest classifying supraventricular and ventricular samples. Thus, this model is selected to be part of the detection component.

## 8. Conclusions

IoT technologies solve problems in various fields such as health. In such a way, the remote monitoring system for cardiac signals, proposed in this work, enables remote supervision providing a support tool in the timely detection of problems related to arrhythmias such as ventricular, supraventricular, and fusion beats and improves medical service and patient's quality of life.

Architectural decisions presented in this work are useful in solving similar problems that require remote supervision of a given variable where IoT technology is suitable. For instance, separate components allow separating responsibilities and using different technologies according to the needs of every component. This approach helps in the decoupling, scalability, and maintenance of the system.

A nonrelational database provides a simple mechanism to store data such as JSON due to the flexibility it provides in the data structure. In addition, API REST simplifies database management providing CRUD operations instead of implementing a database client in every component. In this sense, required changes in the database imply modifications only on the data management component.

On the other hand, it is evident that the KNN algorithm has superior performance over convolutional neural networks and the random forest, in the classification of supraventricular, ventricular, and fusion beats arrhythmias.

## Figures and Tables

**Figure 1:** The 12 lead groups [26].

**Figure 2:** K-nearest neighbors.

**Figure 3:** Random forest [16].

**Figure 4:** System architecture.

**Figure 5:** Training samples distribution.

**Figure 6:** Confusion matrix (CNN).

**Figure 7:** Confusion matrix (random forest).

**Figure 8:** Confusion matrix (KNN).

**Table 1:** Confusion matrix.

		Predicted class	
		Negative	Positive
True class	Negative	TN	FP
	Positive	FN	TP

## Data Availability

All data generated or analyzed during this study are included in the manuscript.
